# A Flexible Extension of Pareto Distribution: Properties and Applications

**DOI:** 10.1155/2021/9819200

**Published:** 2021-08-17

**Authors:** Huda M. Alshanbari, Abd Al-Aziz Hosni El-Bagoury, Ahmed M. Gemeay, E. H. Hafez, Ahmed Sedky Eldeeb

**Affiliations:** ^1^Department of Mathematical Sciences, College of Science, Princess Nourah bint Abdulrahman University, Riyadh, Saudi Arabia; ^2^Department of Mathematics, Faculty of Science, Tanta University, Tanta 31527, Egypt; ^3^Department of Mathematics, Faculty of Science, Helwan University, Helwan, Egypt; ^4^Department of Business Administration, College of Business, King Khaled University, Abha, Saudi Arabia; ^5^Department of Statistics, Mathematics and Insurance, Alexandria University, Alexandria, Egypt

## Abstract

This paper introduced a relatively new mixture distribution that results from a mixture of Fréchet–Weibull and Pareto distributions. Some properties of the new statistical model were derived, such as moments with their related measures, moment generating function, mean residual life function, and mean deviation. Furthermore , different estimation methods were introduced for determining the unknown parameters of the proposed model. Finally, we introduced three real data sets which were applied to our distribution and compared them with other well-known statistical competitive models to show the superiority of our model for fitting the three real data sets, and we can clearly see that our distribution outperforms its competitors. Also, to verify our results, we carried out the existence and uniqueness test to the log-likelihood to determine whether the roots are global maximum or not.

## 1. Introduction

Modeling new phenomena is very important in the field of big data and data science. There are many ways for modeling and representing data. One of these ways is the statistical modeling for real data sets. Statistical modeling is very important in real-life sciences, as many applications and phenomena appear every era of time, so the continuous need for new distribution grows larger. As we know, many of the phenomena that arise nowadays need modeling, but, unfortunately, the traditional distribution could not model them. So, sometimes researchers turn to add new parameters, may be two parameters, to overcome these deficiencies in modeling new phonemes. But there is a new way to overcome all the deficiencies in the traditional distribution.

This method is formulated by making a mixture from two or three distributions to formulate a new superior that can model all the data that the traditional ones failed to model. Many authors worked on the Pareto distribution; see [1], where the authors worked on the Pareto-IV distribution and estimated its parameters under accelerated life test, when the items were under type-II censored sample. Also, as an example for authors that worked on the Fréchet distribution, see [2], where the authors estimated the parameters of the Fréchet distribution under type -II censoring scheme using classical and Bayesian estimation methods.

Mixture distribution may appropriately be utilized for specific data set where various subsets of the entire data set have various properties that can best be demonstrated independently. They can be more mathematically manageable because the individual mixture components deal with that more nicely compared to the overall mixture density. Applications of the mixture of distributions play an important role in reliability theory, insurance risk theory, and the oil industry. Willmot [3] presented the asymptotic tail behavior of Poisson mixtures with applications. Giudici et al. [4] made a novel methodology, dependent on mixtures of the product of Dirichlet process priors, which gave a formal inferential device to think about the logical influence of each covariate.

Without characterizing the system, Bucar et al. [5] demonstrated that the reliability of this system could be approximated by utilizing a finite Weibull mixture distribution. Nakhi and Kalla [6] discussed the mixture of hyper-Poisson distribution with mixing a generalized gamma distribution and hyper-Poisson distribution generalized gamma mixtures.

Panjer and Willmot [7] discover the estimator of the scale parameter in mixture models and the inadmissibility of the unusual estimator set up by displaying better estimators. They used these outcomes in mixtures of normal distributions and mixtures of exponential distributions. Karim et al. [8] introduced Rayleigh mixture distribution with various weight functions, and two correlated Rayleigh random variables have been determined.

By presuming that the random variable *X* has a mixture of distributions if at least one parameter of the distribution of *X* is also a random variable. Let *g*(*x*; *θ*) be probability density function (PDF) of *X*, where *θ* is a parameter of the distribution of *X*. If *θ* is a random variable, then *X* has a mixture of distributions. The PDF of *X* is defined as

(1) $$\begin{array}{c} f\left(x\right)=\left\{\begin{array}{cc} \int_{\theta }g\left(x;\theta \right)h\left(\theta \right)\text{d}\theta , & \theta \text{ is a continuous random variable,}\\ \sum_{\theta }g\left(x;\theta \right)h\left(\theta \right), & \theta \text{ is a discrete random variable.} \end{array}\right) \end{array}$$

Extreme point distributions have developed as one of the most important statistical fields for the applied sciences. Techniques of extreme point are also becoming heavily utilized in many other fields. Extreme point analyses often involve estimate of the likelihood of occurrences which are more extreme than any previously recorded event. Fréchet and Weibull distributions are the most important models for extreme values, and many statisticians have studied these models in many published papers according to their importance in many fields such as earthquakes, floods, engineering, physics, quality control, and medicine. For more information about Fréchet and Weibull distributions, see [1, 2, 9, 10].

So, the main concern of this research is that we derive a mixture distribution called Fréchet–Weibull mixture Pareto distribution (FWMPD) from mixing Fréchet–Weibull distribution with Pareto distribution. This new mixture has a lot of significant advantages, which are very flexible and versatile. This distribution can model skewed and symmetric as well as asymmetric data. Now we will introduce the concept that we based our proposed distribution on.

In order to make the paper easier for the reader, we sectioned and written the paper as follows: In Section 2, we introduce the proposed distribution and the steps to formulate it. In Section 3, we deduce some of the statistical properties of the proposed distribution mathematically. In Section 4, we introduce eight different classical methods for estimating unknown parameters of the proposed model. For more about different kinds of classical methods of estimation, see [11–14] and [15]. In Section 5, we introduce three real data sets as an application to assess the performance of the distribution and to show its efficiency for fitting different real data sets. In Section 6, we introduce the conclusions illustrated from the paper along with the major findings.

## 2. The Mixture of Fréchet–Weibull and Pareto Distributions

The formulation of the new mixture model is presented in this part of the paper . The PDF and the cumulative distribution function (CDF) of the Fréchet–Weibull distribution [16] (*X* > 0) is represented as follows:

(2) $$\begin{array}{c} f\left(x\right)=\alpha k\beta^{\alpha }\lambda^{\alpha k}x^{-1-\alpha k}\exp\left(-\beta^{\alpha }{\left(\frac{\lambda }{x}\right)}^{\alpha k}\right),\\ F\left(x\right)=\exp\left(-\beta^{\alpha }{\left(\frac{\lambda }{x}\right)}^{\alpha k}\right), \end{array}$$

where *α* and *k* are shape parameters and *λ* and *β* are scale parameters.

The PDF and the CDF for the Pareto random variable *X* ≥ *b* are, respectively, given by

(3) $$\begin{array}{c} f\left(x\right)=\frac{ab^{a}}{x^{a+1}},\\ F\left(x\right)=1-{\left(\frac{b}{x}\right)}^{a}, \end{array}$$

where *b* is a scale parameter and *a* is a shape parameter.

If a random variable *X* follows Fréchet–Weibull distribution and by taking one of its four parameters (*λ*) as a random variable following Pareto distribution, then it is said to have FWMPD when its PDF and CDF are, respectively, defined as follows:

(4) $$\begin{array}{c} f\left(x\right)=ab^{a}\beta^{a/k}x^{-a-1}\Gamma \left[1-\frac{a}{k\alpha },\beta^{\alpha }{\left(\frac{b}{x}\right)}^{k\alpha }\right],\;x,a,b,\alpha ,\beta ,k>0, \end{array}$$

(5) $$\begin{array}{c} F\left(x\right)=e^{-\beta^{\alpha }{\left(b/x\right)}^{\alpha k}}-{\left(\frac{b}{x}\right)}^{a}\beta^{a/k}\Gamma \left[1-\frac{a}{k\alpha },\beta^{\alpha }{\left(\frac{b}{x}\right)}^{k\alpha }\right], \end{array}$$

where *a*, *α*, and *k* are shape parameters, *b* and *β* are scale parameters, and Γ[1 − (*a*/*kα*), *β*^*α*^(*b*/*x*)^*kα*^] is upper incomplete gamma function.

### 2.1. Survival and Hazard Functions

The characteristics dependent on the reliability function and its correlated functions are very useful to study the example of any lifetime phenomenon. The survival function [*S*(*x*)], hazard function [*h*(*x*)], and reverse hazard function [*r*(*x*)] of FWMPD are defined as follows:

(6) $$\begin{array}{c} S\left(x\right)=1-e^{-\beta^{\alpha }{\left(b/x\right)}^{\alpha k}}+{\left(\frac{b}{x}\right)}^{a}\beta^{a/k}\Gamma \left[1-\frac{a}{k\alpha },\beta^{\alpha }{\left(\frac{b}{x}\right)}^{k\alpha }\right],\\ h\left(x\right)=\frac{a{\left(b/x\right)}^{a}\beta^{a/k}\Gamma \left[1-\left(a/k\alpha \right),\beta^{\alpha }{\left(b/x\right)}^{k\alpha }\right]}{x\left[{\left(b/x\right)}^{a}\beta^{a/k}\Gamma \left[1-\left(a/k\alpha \right),\beta^{\alpha }{\left(b/x\right)}^{k\alpha }\right]-e^{-\beta^{\alpha }{\left(b/x\right)}^{\alpha k}}+1\right]},\\ r\left(x\right)=\frac{a{\left(b/x\right)}^{a}\beta^{a/k}\Gamma \left[1-\left(a/k\alpha \right),\beta^{\alpha }{\left(b/x\right)}^{k\alpha }\right]}{x\left[e^{-\beta^{\alpha }{\left(b/x\right)}^{ak}}-{\left(b/x\right)}^{a}\beta^{a/k}\Gamma \left[1-\left(a/k\alpha \right),\beta^{\alpha }{\left(b/x\right)}^{k\alpha }\right]\right]}, \end{array}$$

where Γ[1 − (*a*/*kα*), *β*^*α*^(*b*/*x*)^*kα*^] is upper incomplete gamma function.

### 2.2. Asymptotic Behavior

This section contains studies on the behaviors of PDF, CDF, and *S*(*x*) of FWMPD at *x*=0 and *x*=*∞*, respectively, as follows:

(7) $$\begin{array}{c} \underset{x⟶0}{\lim}f\left(x\right)=ab^{a}\beta^{a/k}\underset{x⟶0}{\lim}x^{-a-1}\underset{x⟶0}{\lim}\Gamma \left[1-\frac{a}{k\alpha },\beta^{\alpha }{\left(\frac{b}{x}\right)}^{k\alpha }\right]=ab^{a}\beta^{a/k}\times 0\times 0=0,\\ \underset{x⟶\infty }{\lim}f\left(x\right)=ab^{a}\beta^{a/k}\underset{x⟶\infty }{\lim}x^{-a-1}\underset{x⟶\infty }{\lim}\Gamma \left[1-\frac{a}{k\alpha },\beta^{\alpha }{\left(\frac{b}{x}\right)}^{k\alpha }\right]=ab^{a}\beta^{a/k}\times 0\times \Gamma \left[1-\frac{a}{k\alpha }\right]=0,\\ \underset{x⟶0}{\lim}F\left(x\right)=\underset{x⟶0}{\lim}e^{-\beta^{\alpha }{\left(b/x\right)}^{\alpha k}}-\beta^{a/k}\underset{x⟶0}{\lim}{\left(\frac{b}{x}\right)}^{a}\Gamma \left[1-\frac{a}{k\alpha },\beta^{\alpha }{\left(\frac{b}{x}\right)}^{k\alpha }\right]=0-\beta^{a/k}\times 0=0,\\ \underset{x⟶\infty }{\lim}F\left(x\right)=\underset{x⟶\infty }{\lim}e^{-\beta^{\alpha }{\left(b/x\right)}^{\alpha k}}-\beta^{a/k}\underset{x⟶\infty }{\lim}{\left(\frac{b}{x}\right)}^{a}\Gamma \left[1-\frac{a}{k\alpha },\beta^{\alpha }{\left(\frac{b}{x}\right)}^{k\alpha }\right]=1-\beta^{a/k}\times 0\times \Gamma \left[1-\frac{a}{k\alpha }\right]=1, \end{array}$$

and since *F*(*x*)+*S*(*x*)=1, we have

(8) $$\begin{array}{c} \underset{x⟶0}{\lim}S\left(x\right)=1,\\ \underset{x⟶\infty }{\lim}S\left(x\right)=0. \end{array}$$

### 2.3. Impact of Changing Parameters Values

In this section, we display the impact of changing parameters values on drawing PDF, CDF, *S*(*x*), and *h*(*x*) of FWMPD, which are graphed and plotted in Figures 1–4.

Figure 1(a) explains how the behavior of PDF of FWMPD is affected by increasing the value of parameter *k*, where *α*=0.5, *β*=3, *a*=1.5, and *b*=0.75, and Figure 1(b) explains how its behavior is affected by increasing the value of parameter *β*, where *α*=1, *k*=3, *a*=1.5, and *b*=2.

Figure 2(a) shows how the behavior of CDF is changed when the significance increasing happened of the parameter *a*, as we can see this effect very clearly from the graph, where *α* = 2, *β* = 3, *k* = 0.75, and *b* = 0.5, and Figure 2(b) shows how the behavior of CDF is affected by increasing the value of parameter *b*, where *α* = 0.5, *β* = 0.75, *a* = 1.5, and *k* = 3.

Figure 3(a) shows how the behavior of *S*(*x*)is changed when the significance increasing happened of the parameter *α*, as we can see this effect very clearly from the graph, where *a* = 2, *β* = 0.5, *k* = 0.75, and *b* = 1 are still fixed, and Figure 3(b) shows how the behavior of *S*(*x*) is affected with changing the value of parameter *β*, where *a* = 5, *α* = 3, *k* = 1.5, and *b* = 0.5.

Figure 4(a) shows how the behavior of *h*(*x*) is changed when the significanceincreasing happened of the parameter *k*, as we can see this effect very clearly from the graph, where *a* = 4, *β* = 0.5, *α* = 1, and *b* = 0.75, and Figure 4(b) shows how the behavior of *h*(*x*) is affected by the change of parameter *β*, where *a* = 0.75, *k* = 2, *α* = 3, and *b* = 0.5.

## 3. Statistical Properties

In this part of the paper, we introduce the mathematical properties for the proposed distribution. These properties are the moments, moment generating function, mean residual life function, and the mean deviation of the proposed distribution.

### 3.1. Moments

In this subsection, we present the *r*^*th*^ moments of the proposed distribution. Now let *μ*_*r*_′ be the *r*^*th*^ about the origin of FWMPD and it is defined as follows:

(9) $$\begin{array}{c} \mu_{r}^{\prime }=\int_{x=0}^{\infty }x^{r}f\left(x\right)\text{d}x=\frac{ab^{r}\beta^{r/k}\Gamma \left(1-\left(r/k\alpha \right)\right)}{a-r},\;a>r. \end{array}$$

By setting *r* = 1, 2, 3, and 4, we can get so easily the first four moments by assigning FWMPD, respectively. Therefore, the mean and variance of FWMPD are given by

(10) $$\begin{array}{c} \mu_{1}^{\prime }=\;\mu =\frac{ab\beta^{1/k}\Gamma \left(1-\left(1/k\alpha \right)\right)}{a-1},\\ \sigma^{2}=\frac{ab^{2}\beta^{2/k}\left({\left(a-1\right)}^{2}\Gamma \left(1-\left(2/k\alpha \right)\right)-\left(a-2\right)a\Gamma {\left(1-\left(1/k\alpha \right)\right)}^{2}\right)}{\left(a-2\right){\left(a-1\right)}^{2}}, \end{array}$$

respectively, and, by using the moments about the origin, we can determine the first four central moments about the mean of FWMPD, which are given by the following relations:

(11) $$\begin{array}{c} \mu_{1}=\mu_{1}^{\prime }-\mu =0,\\ \mu_{2}=\mu_{2}^{\prime }-9{\left(\mu_{1}^{\prime }\right)}^{2}=\frac{ab^{2}\beta^{2/k}\left({\left(a-1\right)}^{2}\Gamma \left(1-\left(2/k\alpha \right)\right)-\left(a-2\right)a\Gamma {\left(1-\left(1/k\alpha \right)\right)}^{2}\right)}{\left(a-2\right){\left(a-1\right)}^{2}},\\ \mu_{3}=\mu_{3}^{\prime }-3\;\mu_{2}^{\prime }\mu_{1}^{\prime }+2{\left(\mu_{1}^{\prime }\right)}^{3}=ab^{3}\beta^{3/k}\left(\frac{a\Gamma \left(1-\left(1/k\alpha \right)\right)\left(2a\Gamma {\left(1-\left(1/k\alpha \right)\right)}^{2}-\left(3{\left(a-1\right)}^{2}\Gamma \left(1-\left(2/k\alpha \right)\right)/a-2\right)\right)}{{\left(a-1\right)}^{3}}+\frac{\Gamma \left(1-\left(3/k\alpha \right)\right)}{a-3}\right),\\ \mu_{4}=\mu_{4}^{\prime }-4\;\mu_{3}^{\prime }\mu_{1}^{\prime }+6\;\mu_{2}^{\prime }{\left(\mu_{1}^{\prime }\right)}^{2}-3{\left(\mu_{1}^{\prime }\right)}^{4}=ab^{4}\beta^{4/k}\\ \times \left(\frac{a\Gamma \left(1-\left(1/k\alpha \right)\right)\left(-3a^{2}\Gamma {\left(1-\left(1/k\alpha \right)\right)}^{3}-4{\left(a-1\right)}^{3}\Gamma \left(1-\left(3/k\alpha \right)\right)/a-3+6a{\left(a-1\right)}^{2}\Gamma \left(1-\left(1/k\alpha \right)\right)\Gamma \left(1-\left(2/k\alpha \right)\right)/a-2\right)}{{\left(a-1\right)}^{4}}+\frac{\Gamma \left(1-\left(4/k\alpha \right)\right)}{a-4}\right), \end{array}$$

respectively, which will be used to determine coefficients of skewness, kurtosis, and variation, respectively, as follows:

(12) $$\begin{array}{c} \beta_{1}=\frac{{\left(\mu_{3}\right)}^{2}}{{\left(\mu_{2}\right)}^{3}}=\frac{a-2}{a}\\ \times \frac{{\left(\left(\left(a-2\right){\left(a-1\right)}^{3}/\left(a-3\right)\right)\Gamma \left(1-\left(3/k\alpha \right)\right)-a\Gamma \left(1-\left(1/k\alpha \right)\right)\left(3{\left(a-1\right)}^{2}\Gamma \left(1-\left(2/k\alpha \right)\right)-2\left(a-2\right)a\Gamma {\left(1-\left(1/k\alpha \right)\right)}^{2}\right)\right)}^{2}}{a{\left({\left(a-1\right)}^{2}\Gamma \left(1-\left(2/k\alpha \right)\right)-\left(a-2\right)a\Gamma {\left(1-\left(1/k\alpha \right)\right)}^{2}\right)}^{3}},\\ \beta_{2}=\frac{\mu_{4}}{{\left(\mu_{2}\right)}^{2}}\\ =\frac{{\left(a-2\right)}^{2}{\left(a-1\right)}^{4}\left(\left(a\Gamma \left(1-\left(1/k\alpha \right)\right)\left(-3a^{2}\Gamma {\left(1-\left(1/k\alpha \right)\right)}^{3}-\left(4{\left(a-1\right)}^{3}\Gamma \left(1-\left(3/k\alpha \right)\right)/a-3\right)+\left(6a{\left(a-1\right)}^{2}\Gamma \left(1-\left(1/k\alpha \right)\right)\Gamma \left(1-\left(2/k\alpha \right)\right)/a-2\right)\right)\right)/\left({\left(a-1\right)}^{4}\right)\right)+\left(\Gamma \left(1-\left(4/k\alpha \right)\right)/a-4\right)}{a{\left({\left(a-1\right)}^{2}\Gamma \left(1-\left(2/k\alpha \right)\right)-\left(a-2\right)a\Gamma {\left(1-\left(1/k\alpha \right)\right)}^{2}\right)}^{2}},\\ CV=\frac{\sigma }{\mu }\times 100=\frac{\sqrt{a\left({\left(a-1\right)}^{2}\Gamma \left(1-\left(2/k\alpha \right)\right)-\left(a-2\right)a\Gamma {\left(1-\left(1/k\alpha \right)\right)}^{2}\right)/a-2}}{a\Gamma \left(1-\left(1/k\alpha \right)\right)}. \end{array}$$

### 3.2. Moment Generating Function

The moment generating function of FWMPD is given by

(13) $$\begin{array}{c} M\left(t\right)=ab^{a}\lambda^{-a-1}\sum_{m=0}^{\infty }\frac{t^{m}\lambda^{m}\beta^{m/k}\Gamma \left(1-\left(m/k\alpha \right)\right)}{m!},\;a>m, \end{array}$$

and its characteristic function is given by

(14) $$\begin{array}{c} \phi \left(t\right)=ab^{a}\lambda^{-a-1}\sum_{m=0}^{\infty }\frac{{\left(\text{it}\right)}^{m}\lambda^{m}\beta^{m/k}\Gamma \left(1-\left(m/k\alpha \right)\right)}{m!},\;a>m. \end{array}$$

### 3.3. Mean Residual Life Function

The mean residual life function of a continuous random variable *X* and survival function *S*(*X*) following FWMPD is given by

(15) $$\begin{array}{c} \mu \left(x\right)=E\left(X-x|X>x\right)=\frac{1}{S\left(x\right)}\int_{x}^{\infty }S\left(u\right)\text{d}u=\frac{1}{S\left(x\right)}\int_{x}^{\infty }uf\left(u\right)\text{d}u-x\\ =\;\frac{ab^{a}\beta^{a/k}}{\left(a-1\right)S\left(x\right)}\left[x^{\left(1-a\right)}\Gamma \left(1-\frac{a}{k\alpha },\beta^{\alpha }{\left(\frac{b}{x}\right)}^{k\alpha }\right)+\beta^{1-a/k}b^{1-a}\gamma \left(1-\frac{1}{k\alpha },\beta^{\alpha }{\left(\frac{b}{x}\right)}^{k\alpha }\right)\right]-x,\;a>1, \end{array}$$

where Γ(1 − (*a*/*kα*), *β*^*α*^(*b*/*x*)^*kα*^) and *γ*(1 − (1/*kα*), *β*^*α*^(*b*/*x*)^*kα*^) denote upper and lower in complete gamma function, respectively. We can notice that

(16) $$\begin{array}{c} \mu \left(0\right)=\frac{ab^{a}\beta^{a/k}}{\left(a-1\right)S\left(0\right)}\left[0+\beta^{1-a/k}b^{1-a}\Gamma \left(1-\frac{1}{k\alpha }\right)\right]=\frac{ab\beta^{1/k}\Gamma \left(1-\left(1/k\alpha \right)\right)}{a-1}=E\left(x\right), \end{array}$$

which is an important property for *μ*(*x*).

### 3.4. Mean Deviation

The mean deviation about the mean for FWMPD is given by

(17) $$\begin{array}{c} \text{MD}=\int_{x=0}^{\infty }\left|x-\mu \right|f\left(x\right)\text{d}x=2\;\mu \left(F\left(\mu \right)-1\right)+2\int_{\mu }^{\infty }xf\left(x\right)\text{d}x\\ =2\;\mu \left(F\left(\mu \right)-1\right)+\frac{2ab^{a}\beta^{a/k}}{\left(a-1\right)}\left[\mu^{\left(1-a\right)}\Gamma \left(1-\frac{a}{k\alpha },\beta^{\alpha }{\left(\frac{b}{\mu }\right)}^{k\alpha }\right)+\beta^{1-a/k}b^{1-a}\gamma \left(1-\frac{1}{k\alpha },\beta^{\alpha }{\left(\frac{b}{\mu }\right)}^{k\alpha }\right)\right],\;a>1, \end{array}$$

where Γ(1 − (*a*/*kα*), *β*^*α*^(*b*/*μ*)^*kα*^) and *γ*(1 − 1*k*/*α*, *β*^*α*^(*b*/*μ*)^*kα*^) indicate upper and lower incomplete gamma function, respectively, and, by changing *μ* with any measure of central tendency, we can find its mean deviation.

## 4. Classical Methods of Estimation

This section discusses the conventional techniques for estimating the suggested model parameters *θ*=(*a*, *b*, *α*, *β*, *k*)^⊤^ by eight different classical estimation methods. Many papers discussed these methods (for more information, see [17–21]). Determining the estimated parameters in explicit form is mathematically complicated, so these estimates will be obtained numerically by using Wolfram Mathematica software version 12.0.

### 4.1. Classical Methods for the Complete Sample

In this subsection, we introduce eight methods of estimation which were used for estimating the parameters of the proposed distribution.

#### 4.1.1. Maximum Likelihood Estimates (MLEs)

Let *x*_1_,…, *x*_*n*_ is a randomized sample having a size *n* from the PDF (3). So, the log-likelihood function for *θ* is as follows:

(18) $$\begin{array}{c} \ell =na\;\log\;b+\frac{na\;\log\;\beta }{k}+n\;\log\;a-\left(a+1\right)\sum_{i=1}^{n}\log\;x_{i}+\sum_{i=1}^{n}\log\Gamma \left(1-\frac{a}{k\alpha },\beta^{\alpha }{\left(\frac{b}{x_{i}}\right)}^{k\alpha }\right). \end{array}$$

The MLEs of *θ* can be obtained by maximizing *ℓ*.

#### 4.1.2. Ordinary Least-Squares Estimates (OLSEs)

Let *x*_1:*n*_,…, *x*_*n*:*n*_ be the corresponding order statistics. The OLSEs for the distribution parameters can be easily obtained by making the following equation at minimum value, by using any mathematical software, may be MATHEMATICA 12 or any advanced program.

(19) $$\begin{array}{c} O=\sum_{i=1}^{n}{\left[F\left(x_{i:n}\right)-\frac{i}{n+1}\right]}^{2}=\sum_{i=1}^{n}{\left[e^{-\beta^{\alpha }{\left(b/x_{i:n}\right)}^{\alpha k}}-{\left(\frac{b}{x_{i:n}}\right)}^{a}\beta^{a/k}\Gamma \left[1-\frac{a}{k\alpha },\beta^{\alpha }{\left(\frac{b}{x_{i:n}}\right)}^{k\alpha }\right]-\frac{i}{n+1}\right]}^{2}. \end{array}$$

#### 4.1.3. Weighted Least-Squares Estimates (WLSEs)

By minimizing the following equation, the WLSEs of proposed model parameters can be computed:

(20) $$\begin{array}{c} W=\;\sum_{i=1}^{n}\frac{{\left(n+1\right)}^{2}\left(n+2\right)}{i\left(n-i+1\right)}{\left[F\left(x_{i:n}\right)-\frac{i}{n+1}\right]}^{2}\\ =\sum_{i=1}^{n}\frac{{\left(n+1\right)}^{2}\left(n+2\right)}{i\left(n-i+1\right)}{\left[e^{-\beta^{\alpha }{\left(b/x_{i:n}\right)}^{\alpha k}}-{\left(\frac{b}{x_{i:n}}\right)}^{a}\beta^{a/k}\Gamma \left[1-\frac{a}{k\alpha },\beta^{\alpha }{\left(\frac{b}{x_{i:n}}\right)}^{k\alpha }\right]-\frac{i}{n+1}\right]}^{2}. \end{array}$$

#### 4.1.4. Anderson–Darling Estimates (ADEs), Right-Tail Anderson–Darling Estimates (RTADEs), and Left-Tail Anderson–Darling Estimates (LTADEs)

The ADEs for the distribution parameters can be easily obtained by making the following equation at minimum value, by using any mathematical software, may be MATHEMATICA 12 or any advanced program.

(21) $$\begin{array}{c} A=-n-\frac{1}{n}\sum_{i=1}^{n}\left(2i-1\right)\left[\log\;F\left(x_{i:n}\right)+\log\;S\left(x_{i:n}\right)\right]. \end{array}$$

The RTADEs for the distribution parameters can be easily obtained by making the following equation at minimum value, by using any mathematical software, may be MATHEMATICA 12 or any advanced program.

(22) $$\begin{array}{c} R=\frac{n}{2}-2\sum_{i=1}^{n}F\left(x_{i:n}\right)-\frac{1}{n}\sum_{i=1}^{n}\left(2i-1\right)\log\;S\left(x_{i:n}\right). \end{array}$$

The LTADEs for the distribution parameters can be easily obtaine by making the following equation at minimum value, by using any mathematical software, may be MATHEMATICA 12 or any advanced program.

(23) $$\begin{array}{c} L=-\frac{3}{2}n+2\sum_{i=1}^{n}F\left(x_{i:n}\right)-\frac{1}{n}\sum_{i=1}^{n}\left(2i-1\right)\log\;F\left(x_{i:n}\right). \end{array}$$

#### 4.1.5. Cramér–von Mises Estimates (CVMEs) and Maximum Product of Spacing Estimates (MPSEs)

The CVMEs are determined by minimizing

(24) $$\begin{array}{c} \text{CV}=\frac{1}{12n}+\sum_{i=1}^{n}{\left[F\left(x_{i:n}\right)-\frac{2i-1}{2n}\right]}^{2}\\ \;=\frac{1}{12n}+\sum_{i=1}^{n}{\left[e^{-\beta^{\alpha }{\left(b/x_{i:n}\right)}^{\alpha k}}-{\left(\frac{b}{x_{i:n}}\right)}^{a}\beta^{a/k}\Gamma \left[1-\frac{a}{k\alpha },\beta^{\alpha }{\left(\frac{b}{x_{i:n}}\right)}^{k\alpha }\right]-\frac{2i-1}{2n}\right]}^{2}. \end{array}$$

The MPSEs are determining by maximizing the following equation:

(25) $$\begin{array}{c} G=\frac{1}{n+1}\sum_{i=1}^{n+1}\log\left(D_{i}\right), \end{array}$$

where *D*_*i*_=*F*(*x*_*i*_) − *F*(*x*_*i*−1_), *F*(*x*_0_)=0, *F*(*x*_*n*+1_=1), and ∑_*i*=1_^*n*+1^*D*_*i*_=1.

## 5. Modeling Real Data Sets

This section discusses the flexibility of the proposed model for fitting three real-world data sets and compares it with other well-known competing models. The three analyzed data sets are used to show the flexibility of FWMED as we used very common distribution for comparison that they are known by their flexibility such as Fréchet–Weibull mixture exponential distribution (FWMED) [22], Weibull distribution (WD), exponential distribution (ED), gamma distribution (GD), and inverse Pareto distribution (IPD) [23].

The competing distributions are compared using goodness-of-fit measures, including Anderson–Darling (AD), Cramér–von Mises (CM), and Kolmogorov–Smirnov (KS) with its *p* value (KS-*p* value).

To evaluate the validity of competing models, the MLEs method is used for esitimatingthe parameters of the competing models, and the analytical measurements are generated using the Wolfram Mathematica version 12 program. 

### 5.1. Data Set I

This real data set is for the relief times of twenty patients taking a acertain kind of medecine called analgesic. These data were introduced by Clark and Gross [24], page 105, and they are given in Table 1.

Table 2 provides the analytical measures along with MLEs. The fitted PDF, CDF, SF, and P-P plots of the FWMPD model for the first data set are depicted in Figure 5. The results in Table 2 show that the FWMPD distribution is the best fit one compared to other models that are comparable for the first data set.  Figure 6 provides profile-likelihood plots of the FWMPD parameters for the first real data set. These plots illustrate the unimodality of profile-likelihood functions for all estimated parameters.  Table 3 presents the values of estimates, negative log-likelihood function, CM, AD, KS, and KSP of the proposed model for the eight different estimation methods.  Figure 7 displays P-P plots for the proposed model by using different estimation methods along with fitted PDFs by results of these methods.

### 5.2. Data Set II

This data set was taken from McCool, and it represents the fatigue lifetime in hours for 10 bearings of certain types. It was studied by Wu and Wong [25], and it is given in Table 4.

Table 5 provides the analytical measures along with ML estimates. The fitted PDF, CDF, SF, and P-P plots of the FWMPD model for the second data set are depicted in Figure 8. The results in Table 5 show that the FWMPD distribution is the best fit compared to other models that are comparable for the second data set.  Figure 9 provides the profile-likelihood plots of the FWMPD parameters for the second real data set. These plots illustrate the unimodality of profile-likelihood functions for all estimated parameters.  Table 6 presents the values of estimates, negative log-likelihood function, CM, AD, KS, and KSP of the proposed model for the eight different estimation methods.  Figure 10 displays the P-P plots for the proposed model by using different estimation methods along with fitted PDFs by results of these methods.

### 5.3. Data Set III

This data set indicates the survival times for head neck cancer of 45 patients; we consider this data set as a complete one. For more details about the data, see [26]. This data set is given in Table 7.  Table 8 provides the analytical measures along with ML estimates. The fitted PDF, CDF, SF, and P-P plots of the FWMPD model for the third data set are depicted in Figure 11. The results in Table 8 show that the FWMPD distribution is the best fit compared to other models that are comparable for the third data set.  Figure 12 provides profile-likelihood plots of the FWMPD parameters for the third real data set. These plots illustrate the unimodality of profile-likelihood functions for all estimated parameters.  Table 9 presents the values of estimates, negative log-likelihood function, CM, AD, KS, and KSP of the proposed model for the eight different estimation methods.  Figure 13 displays P-P plots for the proposed model by using different estimation methods along with fitted PDFs by results of these methods.

### 5.4. Concluding Remarks on the Results of the Real Data Sets

1. Regarding the data sets in Tables 1, 4, and, 7, we applied three data sets to the proposed distribution, and we deduced that the distribution outperforms all its competitors.
2. Referring to the values of the KS, AD, and CM, we can deduce that the proposed distribution has the least measures, and this assures its superiority.
3. Referring to the *P* values of the distribution, we can deduce that the proposed distribution has the highest value, and this assures its superiority.
4. Figures 6, 9, and 12 provide profile-likelihood plots of the FWMPD parameters for the three real data sets, respectively. These plots illustrate that the estimated parameters give a maximum value of the log-likelihood function, and these estimates are global maximum estimates.

## 6. Conclusion and Major Findings

In this article, we introduced a new mixture of distribution FWMPD, and we estimated its parameters by the classical methods of estimation: the maximum likelihood estimation and 7 other methods. We introduced its mathematical properties and graphed its PDF and CDF to study its behavior under different values of estimates. Last but not least, we made an application on the proposed distribution to assure its superiority compared to its competitors. We evaluated its KS, AD, CM, and *P* value, and we deduced that it has the lowest values for KS, AD, and CM and the greatest values for *P* values which make it a better candidate among all its competitors. Also, to make sure that the roots for the MLEs for the proposed distribution give a maximum value, we graphed Figures 6, 9, and 12 for the profile-likelihood function of the proposed model with its parameters for the three real data sets, respectively. These plots illustrate the unimodality of profile-likelihood functions for all estimated parameters. We expect that the presented model will find a broader range of applications in fields like engineering, survival and lifespan data, meteorology, hydrology, and economics.

## Figures and Tables

**Figure 1:** The effects of parameters *k* and *β* on the PDF of FWMPD.

**Figure 2:** The effects of parameters *a* and *b* on the CDF of FWMPD.

**Figure 3:** The effects of parameters *α* and *β* on *S*(*x*) of FWMPD.

**Figure 4:** The effects of parameters *k* and *β* on *h*(*x*) of FWMPD.

**Figure 5:** The fitted FWMPD PDF, CDF, SF, and P-P plots for the first data set. (a–d) FWMPD.

**Figure 6:** Plots of the profile-likelihood functions for the proposed model's MLEs of the first data set.

**Figure 7:** The probability-probability (P-P) plot and the fitted PDFs of the proposed model for the first data set.

**Figure 8:** The fitted FWMPD PDF, CDF, SF, and P-P plots for the second data set. (a–d) FWMPD.

**Figure 9:** Plots of the profile-likelihood functions for the proposed model's MLEs of the second data set.

**Figure 10:** The probability-probability (P-P) plot and the fitted PDFs of the proposed model for the second data set.

**Figure 11:** The fitted FWMPD PDF, CDF, SF, and P-P plots for the third data set. (a–d) FWMPD.

**Figure 12:** Plots of the profile-likelihood functions for the proposed model MLEs of the third data set.

**Figure 13:** The probability-probability (P-P) plot and the fitted PDFs of the proposed model for the third data set.

**Table 1:** Numerical values of the first data set.

1.1	1.4	1.3	1.7	1.9	1.8	1.6	2.2	1.7	2.7
4.1	1.8	1.5	1.2	1.4	3	1.7	2.3	1.6	2

**Table 2:** Goodness-of-fit measures and estimates of FWMPD and other fitted models for the first data set.

Model	AD	CM	KS	KSP	Estimates
FWMPD	0.159942	0.027555	0.101977	0.985411	$\hat{\alpha }=8.26658$
					$\hat{\beta }=1.9737$
					$\hat{k}=0.62992$
					$\hat{a}=5.07903$
					$\hat{b}=0.45048$

FWMED	0.273164	0.034323	0.110737	0.966914	$\hat{\alpha }=1.35077$
					$\hat{a}=3.04669$
					$\hat{\lambda }=2.11748$
					$\hat{k}=4.3601$

ED	4.6035	0.962967	0.439513	0.00088	$\hat{\alpha }=0.526317$

ExED	0.31046	0.047659	0.134314	0.863396	$\hat{\alpha }=36.6832$
					$\hat{a}=2.23524$

WD	1.08354	0.18343	0.18497	0.50057	$\hat{a}=2.78703$
					$\hat{b}=2.12998$

GD	0.59902	0.10251	0.173406	0.584477	$\hat{\alpha }=9.66948$
					$\hat{\lambda }=0.19649$

IPD	4.80207	0.98722	0.38723	0.00496	$\hat{\alpha }=139428$
					$\hat{\theta }=0.000012$

**Table 3:** The estimates and log-likelihood function of the proposed distribution parameters along with goodness-of-fit measures for the first data set by different estimation methods.

	$\hat{\alpha }$	$\hat{\beta }$	$\hat{k}$	$\hat{a}$	$\hat{b}$	−L	AD	CM	KS	KSP
MLEs	8.26658	1.9737	0.629929	5.07903	0.450483	15.3986	0.159942	0.0275557	0.101977	0.985411
ADEs	3.66431	0.427879	1.43692	4.91413	2.38647	15.4012	0.160271	0.0276845	0.100069	0.988169
CVMEs	3.9903	0.390447	1.40609	5.43643	2.63528	15.543	0.195929	0.0252485	0.0932922	0.99498
MPSEs	2.70565	1.1713	1.56485	4.8245	1.17775	15.543	0.195929	0.0252485	0.0932922	0.99498
OLSEs	2.62302	0.441688	1.96049	4.78627	1.99296	15.4157	0.163091	0.0296234	0.101826	0.985646
RTADEs	2.60132	0.847394	1.52364	3.42267	1.39021	16.896	0.605671	0.109102	0.149826	0.760347
WLSEs	2.47207	0.527218	1.17467	2.86848	2.03735	19.8185	1.3916	0.246237	0.203642	0.378108
LTADEs	3.46508	1.46402	1.45574	5.03363	1.02091	15.4074	0.161581	0.0289918	0.097162	0.991618

**Table 4:** The second data set's statistical analysis.

152.7	172.0	172.5	173.3	193.0	204.7	216.5	234.9	262.6	422.6

**Table 5:** Goodness-of-fit measures and estimates of FWMPD and other fitted models for the second data set.

Model	AD	CM	KS	KSP	Estimates
FWMPD	0.203151	0.0281603	0.142074	0.987635	$\hat{\alpha }=22.8864$
					$\hat{\beta }=12.5295$
					$\hat{k}=0.773245$
					$\hat{a}=3.5865$
					$\hat{b}=5.87626$

FWMED	2.7067	0.550077	0.449194	0.0353535	$\hat{\alpha }=1.13686$
					$\hat{a}=0.000914$
					$\hat{\lambda }=0.107839$
					$\hat{k}=0.823594$

ED	2.58977	0.550784	0.499695	0.0135584	$\hat{\alpha }=0.004535$

ExED	0.451539	0.052846	0.185038	0.883325	$\hat{\alpha }=88.952$
					$\hat{a}=0.023466$

WD	0.948293	0.154708	0.219376	0.721648	$\hat{a}=2.93592$
					$\hat{b}=246.409$

GD	0.681532	0.098772	0.185398	0.881913	$\hat{\alpha }=11.5632$
					$\hat{\lambda }=19.0674$

IPD	2.72548	0.565404	0.439931	0.0416838	$\hat{\alpha }=114313$
					$\hat{\theta }=0.0017835$

**Table 6:** The estimates and log-likelihood function of the proposed distribution parameters along with goodness-of-fit measures for the second data set by different estimation methods.

	$\hat{\alpha }$	$\hat{\beta }$	$\hat{k}$	$\hat{a}$	$\hat{b}$	−L	AD	CM	KS	KSP
MLEs	22.8901	12.5283	0.773162	3.58645	5.87487	52.7057	0.203153	0.0281606	0.142078	0.987631
ADEs	10.3482	40.9592	1.29155	3.62364	8.67465	52.7803	0.189819	0.0275719	0.144604	0.984983
CVMEs	8.44699	39.0844	1.23963	4.19593	8.09549	52.8688	0.199311	0.0269341	0.146773	0.982409
MPSEs	10.9242	26.4012	1.18944	2.83251	9.41679	52.8688	0.199311	0.0269341	0.146773	0.982409
OLSEs	22.8901	12.5283	0.775023	3.58651	5.8748	52.7226	0.206266	0.0304352	0.1596527	0.960749
RTADEs	12.7429	46.3221	1.39524	3.47163	9.85431	52.7104	0.198978	0.0281769	0.143302	0.986394
WLSEs	8.12391	46.4511	1.44475	3.18893	10.4892	53.1035	0.22902	0.0344934	0.166636	0.944053
LTADEs	20.9614	43.2579	0.4669297	4.49099	0.0491646	52.9121	0.20854	0.027048	0.149197	0.979187

**Table 7:** Numerical values of the third data set.

37	84	92	94	110	112	119	127	130	133
140	146	155	159	169	173	179	194	195	209
249	281	319	339	432	469	519	528	547	613
633	725	759	817	1092	1245	1331	1557	1642	1771
1776	1897	2023	2146	2297					

**Table 8:** Goodness-of-fit measures and estimates of FWMPD and other fitted models for the third data set.

Model	AD	CM	KS	KSP	Estimates
FWMPD	0.639363	0.084663	0.096699	0.794056	$\hat{\alpha }=10.7787$
					$\hat{\beta }=6.99619$
					$\hat{k}=0.123512$
					$\hat{a}=1.32604$
					$\hat{b}=0.000016$

FWMED	1.01488	0.152155	0.131286	0.419929	$\hat{\alpha }=1.55186$
					$\hat{a}=0.00109$
					$\hat{\lambda }=3.91053$
					$\hat{k}=0.976671$

ED	1.48253	0.241153	0.165597	0.169403	$\hat{\alpha }=0.001564$

ExED	1.58344	0.262442	0.173083	0.134882	$\hat{\alpha }=1.03827$
					$\hat{a}=0.001603$

WD	1.38913	0.220213	0.157802	0.212421	$\hat{a}=0.979504$
					$\hat{b}=632.973$

GD	1.55782	0.257197	0.171239	0.142806	$\hat{\alpha }=1.02661$
					$\hat{\lambda }=622.634$

IPD	0.65175	0.0869602	0.098414	0.776073	$\hat{\alpha }=45.269$
					$\hat{\theta }=4.91826$

**Table 9:** The estimates and log-likelihood function of the proposed distribution parameters along with goodness-of-fit measures for the third data set by different estimation methods.

	$\hat{\alpha }$	$\hat{\beta }$	$\hat{k}$	$\hat{a}$	$\hat{b}$	−L	AD	CM	KS	KSP
MLEs	10.7787	6.99619	0.123512	1.32604	0.00001628	333.508	0.670616	0.09208357	0.0911992	0.848307
ADEs	3.77138	5.37446	0.37446	1.07062	1.14398	333.824	0.635178	0.079101	0.0953321	0.808067
CVMEs	6.3231	4.02213	0.274373	0.82339	0.546817	334.757	0.677278	0.0751701	0.111228	0.633673
MPSEs	3.03965	4.29119	0.412976	1.21881	3.029	334.757	0.677278	0.0751701	0.111228	0.633673
OLSEs	4.87073	4.12184	0.358181	0.784352	1.60477	334.977	0.71475	0.0765975	0.11767	0.561555
RTADEs	4.34644	5.32808	0.29679	1.26154	0.40316	333.589	0.637697	0.0832888	0.0970136	0.790793
WLSEs	3.771387	5.37446	0.37446	1.07062	1.14398	333.824	0.635178	0.07910097	0.0953316	0.808072
LTADEs	2.99381	12.5628	0.57333	0.865617	1.09981	334.578	0.657612	0.0763929	0.105159	0.702176

## Data Availability

All data are included within the paper.
